This article has been retracted.

# Effect of Oral Tranexamic Acid on the Blood Transfusion Rate and the Incidence of Deep Vein Thromboembolism in Patients after TKA

**DOI:** 10.1155/2022/6041827

**Published:** 2022-07-08

**Authors:** Bingqian Chen, Xiaohong Qu, Xiaowen Fang, Xuesong Wang, Guoxiu Ke

**Affiliations:** ^1^Department of Orthopedics, Changshu Hospital, Soochow University, First People's Hospital of Changshu City, Changshu, Jiangsu, China; ^3^Department of Geriatrics, Changshu Hospital, Soochow University, First People's Hospital of Changshu City, Changshu, Jiangsu, China; ^2^Department of Orthopedics, Affiliated Hospital of Jiangnan University, Wuxi, Jiangsu, China

## Abstract

**Purpose:**

To explore the effect of oral tranexamic acid treatment on the blood transfusion rate and the incidence of deep vein thromboembolism after total knee arthroplasty (TKA).

**Methods:**

90 patients undergoing TKA admitted to First People's Hospital of Changshu City from January 2019 to January 2020 were selected and randomized into the control group and the experimental group accordingly (45 cases in each group). The control group intravenously received 20 mL/kg tranexamic acid before the incision was closed. The experimental group was given 1 g of tranexamic acid orally before anesthesia, 6 h and 12 h after the operation.

**Results:**

The experimental group witnessed better perioperative indexes in relation to the control group. The experimental group displayed better postoperative coagulation function indexes as compared to the control group (*P* < 0.05). Remarkably lower postoperative vascular endothelial function indexes in the experimental group than in the control group were observed. The experimental group experienced a markedly lower incidence of deep vein thromboembolism in comparison with the control group (*P* < 0.05). The postoperative knee society score (KSS) score of the experimental group was significantly higher than that of the control group. A significantly higher postoperative modified rivermead mobility index (MRMI) score was yielded in the experimental group in contrast to the control group (*P* < 0.05). The experimental group obtained lower numerical rating scale (NRS) scores at T2 and T3 as compared to the control group.

**Conclusion:**

Oral tranexamic acid is a suitable alternative for patients undergoing TKA in terms of reducing the blood transfusion rate, relieving pain, and accelerating the recovery of the patient's limbs.

## 1. Introduction

The knee joint is considered the most critical lower limb weight-bearing joint in the human body, and its function and structure are the most complicated [1]. Clinically, knee degenerative bone and joint disease is a commonly seen disease, with a prevalence of 34% in the male population over 50 years old and 73% in females [2–4]. Knee degenerative bone and joint disease belong to the category of “arthritis” in traditional Chinese medicine (TCM). TCM believes that this disease is mostly caused by deficiency of liver and kidney, lack of qi and blood, malnutrition of muscles and bones, as well as external pathogens such as cold, dampness, phlegm and blood stasis, or overwork, falling and fluttering, blood stasis, and meridian stasis. TCM treatment methods include external application of knee drugs, oral administration of TCM, acupuncture treatment, small needle knife treatment, knee massage treatment, etc. TCM treatment is recommended for early knee degeneration.

For patients with poor response to conservative treatment, total knee arthroplasty (TKA) is the mainstay for the clinical treatment of this disease, which aims to relieve the patient's pain and restore the patient's knee by replacing the artificial joint with the patient's articular surface damaged by the injury or disease through surgery [5, 6]. To date, the TKA has produced a prominent outcome and is extensively recognized in the clinic setting. Nevertheless, it is associated with large local wounds and a prolonged healing process due to a volume of blood transfusion after surgery, thereby increasing the risk of deep vein thromboembolism and seriously compromising the prognosis of patients. Some scholars have found that the application of tranexamic acid to patients undergoing TKA can effectively reduce postoperative bleeding and reduce the risk of postoperative complications [7–9]. With this background, the present study was conducted to further explore the effect of oral tranexamic acid treatment on the blood transfusion rate and the incidence of deep vein thromboembolism in patients after TKA.

## 2. Materials and Methods

### 2.1. Baseline Information

Altogether, 90 patients undergoing TKA admitted to First People's Hospital of Changshu City from January 2019 to January 2020 were selected and randomized into the control group and the experimental group accordingly (45 cases in each group). This study was approved by the hospital ethics committee, and the patient and his family members were informed of the purpose and process of the trial and signed informed consent. This study complied with the Declaration of Helsinki.

### 2.2. Inclusion and Exclusion Criteria

#### 2.2.1. Inclusion criteria

① age 18∼65 years old; ② in line with TKA treatment indications; ③ with normal preoperative coagulation indexes and blood routine; ④ with unilateral lesions; and ⑤ ineffective or recurrent after conservative treatment.

#### 2.2.2. Exclusion criteria

① with fracture of lower limb; ② patients who has a recent use of anticoagulant drugs within 7 days; ③ patients with coagulation dysfunction; ④ pregnant or lactating women; and ⑤ patients with mental disorders.

### 2.3. Methods

Both groups of patients were treated with TKA via the medial parapatella. First, the patient was given epidural anesthesia, and the tourniquet was tied to the affected limb before the skin incision; a median incision was made in front of the knee joint, and then the surgeon entered the joint cavity from the inside of the parapatella, turned the patella outward, and performed standard osteotomy of the tibial plateau and distal femur. Next, they loosened the soft tissues, balanced the medial and lateral gaps with flexion and extension, and fixed the tibial and femoral prostheses.They also installed a polyethylene gasket to correct the surface of the patella and placed a drainage tube in the posterior joint cavity. After the operation was completed, the loosened tourniquet was pressure-wrapped with cotton pads and elastic bandages.

In the control group, 20 mL/kg tranexamic acid was injected intravenously before the incision was closed (manufacturer: Chongqing Laimei Pharmaceutical Co., Ltd.; approval no.: H20056600; specification: 5 ml: 0.25 g). In the experimental group, 1 g of tranexamic acid was orally administered before anesthesia, 6 h and 12 h after operation (manufacturer: Chongqing Yaoyou Pharmaceutical Co., Ltd.; approval no.: J20160092; specification: 500 mg ^*∗*^20 tablets). The research flow chart is shown in Figure 1.

### 2.4. Outcome Measures

The perioperative indicators including transfusion rate, intraoperative blood transfusion, postoperative blood transfusion, and hidden blood loss were compared. Among them, intraoperative blood transfusion = the amount of fluid in the suction bottle + the net increase of the surgical dressing—the amount of irrigation fluid used during the operation; postoperative blood loss = the amount of wound drainage fluid; hidden blood loss = theoretical total blood loss (preoperative blood volume ^*∗*^(preoperative hematocrit—postoperative hematocrit)) + blood transfusion—blood loss.

The fasting venous blood of the two groups of patients before and after the operation was collected and centrifuged to obtain the plasma. The automatic blood coagulation analyzer was used to detect fibrinogen (Fig), prothrombin time (PT), and activated partial thromboplastin time (APTT).

3 mL of fasting venous blood was collected before and after the operation of the two groups of patients and centrifuged to isolate the serum and placed at −20°C for use. The automatic biochemical detector was used to detect soluble thrombomodulin (sTM), vascular endothelial growth factor (VEGF), and E-selectin in the vascular endothelial function.

The incidence of deep vein thromboembolism in the two groups was compared.

The Keen Society Score (KSS) [10] was used to evaluate the knee joint recovery of the two groups of patients before and after surgery. The scale includes clinical scores and functional scores, both with a total score of 100 points. A higher score suggests better recovery of postoperative knee joints.

The modified rivermead mobility index (MRMI) [11] was adopted to evaluate the patient's limb mobility before and after surgery. The total score is 20 points; the higher the score, the better the patient's limb mobility.

The numerical rating scale [12] was used to evaluate the pain levels of the two groups of patients before surgery, and 12 h, 24 h, and 48 h after surgery. The total score of the scale is 10 points. A higher score indicates more intense pain. T0, T1, T2, and T3 are respectively interpreted as the time points before the operation, 2 h after the operation, 12 h after the operation, and 24 h after the operation.

### 2.5. Statistical Analysis

The software SPSS20.0 was used for data analysis, and GraphPad Prism 7 (GraphPad Software, San Diego, USA) for graphic plotting. The study includes count data and measurement data, which were examined by using the chi-square test, *t*-test, and normality test. A *P* value of 0.05 or lower was taken as the level of significance.

## 3. Results

### 3.1. Comparison of General Information

The two groups did not differ in terms of gender, average age, BMI, average course of disease, operation time, SAS score, SDS score, and place of residence (*P* > 0.05, Table 1).

### 3.2. Comparison of Perioperative Indicators

The experimental group has more favorable perioperative indexes relative to the control group (*P* < 0.05), as shown in Table 2.

### 3.3. Comparison of Coagulation Function Indexes

The experimental group displayed better postoperative coagulation function indexes as compared to the control group (*P* < 0.05, Table 3).

### 3.4. Comparison of Vascular Endothelial Function Indexes

Significantly lower postoperative vascular endothelial function indexes in the experimental group than the control group were observed (*P* < 0.05), see Table 4.

### 3.5. Comparison of the Incidence of Deep Vein Thromboembolism between the Two Groups

In the experimental group, the incidence of postoperative deep vein thromboembolism was 2.22% (2/45) compared to 20.00% (9/45) in the control group. The experimental group experienced a markedly lower incidence of deep vein thromboembolism in comparison with the control group (*P* < 0.05).

### 3.6. Comparison of KSS, MRMI, and NRS Scores

The postoperative KSS score and MRMI score of the experimental group were significantly higher than those of the control group (both *P* < 0.05), as shown in Figure 2.

### 3.7. Comparison of NRS Scores

The experimental group had lower NRS scores at T2 and T3 as compared to the control group (*P* < 0.05) as shown in Figure 3.

## 4. Discussion

As the major approach for clinical treatment of various knee joint diseases, TKA can effectively mitigate the clinical symptoms of patients [13, 14]. It is reported that there are annually 190,000 patients receiving TKA treatment in China, and the figure shows a rising trend [15, 16]. Although effective in correcting patients' joint deformities in the short-term, this approach removes more bones and dissects more tissues during surgery, which is prone to adverse events such as massive bleeding, and is not conducive to the prognosis of patients [17–19]. In order to reduce the perioperative blood loss and the side events caused by blood transfusion, a tourniquet is frequently used in clinical TKA treatment. However, a small number of patients experience abnormal blood coagulation after the tourniquet is released, and the vulnerability to postoperative complications is high [20, 21]. On top of this, some patients are susceptible to ischemia-reperfusion injury after the release of the tourniquet, seriously compromising the prognosis of the patients. Therefore, how to reduce the massive bleeding during the perioperative period of TKA has been a pressing issue among scholars [22]. Additionally, most scholars believe that the reduction of the perioperative bleeding rate in TKA treatment has a positive role in the recovery of patients' physical functions. Tranexamic acid, also known as tranexamic acid, is one of the most widely used anticoagulant drugs in clinical applications. Similar to aminomethylbenzoic acid, it prevents plasminogen from being converted into plasmin, inhibits the proteolytic activity of fibrinolysis, and competes against plasmin activator [23]. As per our knowledge, tranexamic acid is not only suitable for various bleeding caused by hyperfibrinolysis but also for organ trauma or bleeding prevention before surgery with plasminogen activating substances.

Remarkably, the current study found that the perioperative indicators of the experimental group were significantly better than those of the control group, indicating that compared with intravenous infusion, oral tranexamic acid can effectively reduce the patient's perioperative blood transfusion rate. APTT is currently a common and clinically sensitive test to screen whether the endogenous coagulation system is normal, and it is also an important indicator of the activity of coagulation factors VIII, I and IX. As previously noted, PT is a key index that reflects the exogenous coagulation pathway, which can demonstrate the activity of the patient's own coagulation factors. Fig is a kind of fibrinogen, and the abnormality of its index would result in the disorder of blood coagulation [24]. Encouragingly, this study revealed that the experimental group exhibited superior postoperative coagulation function indexes relative to the control group, suggesting that oral tranexamic acid has a milder impact on coagulation function. Moreover, the stress injury during the TKA operation can lead to vascular endothelial cell dysfunction, which coupled with the poor blood circulation of the affected limb after the operation easily results in hypercoagulability, thereby raising the risk of deep vein thromboembolism in patients. In this study, the postoperative vascular endothelial function indexes of the experimental group were significantly lower than those of the control group, indicating that oral tranexamic acid can effectively protect the patient's vascular endothelial cells and reduce postoperative complications. Additionally, the results of the present study showed that the postoperative KSS score and MRMI score of the experimental group were significantly higher than those of the control group, and the NRS scores of the experimental group at T2 and T3 were significantly lower than those of the control group. This finding would suggest that oral administration of tranexamic acid can effectively reduce the pain of patients and accelerate the mobility recovery of knee joints and limbs. Also, we found that the incidence of deep vein thromboembolism in the experimental group was significantly lower than that in the control group, which was in line with the results of the study by Vivekanand et al. [25], who argued that the incidence of deep vein thromboembolism in the observation group was 1.82%, significantly lower than the 14.55% in the control group. It further confirms the safety profile of oral tranexamic acid.

## 5. Conclusion

Oral tranexamic acid is a suitable alternative for patients undergoing TKA by reducing the blood transfusion rate, relieving pain, and accelerating the recovery of the patient's limbs. It is worthy, therefore, of promotion and application.

## Figures and Tables

**Figure 1:** Experimental flowchart.

**Figure 2:** Comparison of KSS and MRMI scores, ^*∗∗∗*^indicated *P* < 0.001.

**Figure 3:** Comparison of NRS scores. Note: The abscissa represents the time points of T0, T1, T2, and T3, and the ordinate represents the NRS score, points. The NRS scores of patients in the experimental group at T0, T1, T2, and T3 were (8.79 ± 1.14), (7.01 ± 0.75), (3.71 ± 0.42), and (1.02 ± 0.11) points, respectively. The NRS scores of patients in the control group at T0, T1, T2, and T3 were (8.78 ± 1.15), (7.11 ± 0.89), (5.88 ± 0.66), and (3.57 ± 0.52) points, respectively. ^*∗*^indicates that there is a significant difference in the NRS score at T2 between the two groups of patients (*t* = 18.608, *P* < 0.001). ^*∗∗*^indicates that there is a significant difference in the NRS score at T3 between the two groups (*t* = 32.184, *P* < 0.001).

**Table 1:** Comparison of general information.

	Experimental group (*n* = 45)	Control group (*n* = 45)	*χ* ^2^/*t*	*P*
Gender			0.055	0.814
Male	13 (28.89)	12 (26.67)		
Female	27 (60.00)	28 (62.22)		
Age (year)	55.25 ± 3.32	55.33 ± 3.29	0.115	0.909
BMI (kg/m2)	26.27 ± 1.59	25.89 ± 1.63	1.119	0.266
Course of disease (year)	6.21 ± 2.17	6.25 ± 2.15	0.088	0.930
Operation time (min)	101.23 ± 13.35	101.31 ± 13.27	0.029	0.978
SAS score	35.22 ± 2.31	35.23 ± 2.27	0.041	0.967
SDS score	45.15 ± 2.31	45.17 ± 2.29	0.041	0.967
Place of residence			0.050	0.822
Town	31 (68.89)	30 (66.67)		
Rural area	14 (31.11)	15 (33.33)		

**Table 2:** Comparison of perioperative indexes.

Groups	n	Postoperative blood transfusion rate (%)	Intraoperative blood transfusion (mL)	Postoperative blood transfusion (mL)	Hidden blood loss (mL)
Experimental group	45	33.33% (15/45)	161.22 ± 31.02	369.25 ± 75.36	527.41 ± 158.35
Control group	45	66.67% (30/45)	182.35 ± 35.27	420.18 ± 111.39	691.85 ± 179.52
*χ* ^2^/*t*		10.000	3.018	2.539	4.608
*P*		<0.05	<0.05	<0.05	<0.001

**Table 3:** Comparison of coagulation function indexes ($\bar{x}$ ± *s*).

Groups	n	Fig (g/L)		PT (s)		APTT (s)	
		Before	After	Before	After	Before	After
Experimental group	45	2.31 ± 0.43	5.11 ± 0.53	11.02 ± 0.38	9.41 ± 1.62	20.38 ± 2.11	24.12 ± 2.29
Control group	45	2.32 ± 0.47	2.98 ± 0.35	11.05 ± 0.35	13.56 ± 1.21	20.27 ± 2.05	27.75 ± 1.77
*t*		0.105	22.497	0.389	13.768	0.251	8.413
*P*		0.916	<0.001	0.698	<0.001	0.803	<0.001

**Table 4:** Comparison of vascular endothelial function indexes ($\bar{x}$ ± *s*, *μ*g/L).

Groups	n	sTM		VEGF		E-Selectin	
		Before operation	After operation	Before operation	After operation	Before operation	After operation
Experimental group	45	5.11 ± 0.35	4.35 ± 0.21	44.27 ± 0.81	35.82 ± 0.34	92.86 ± 0.73	85.36 ± 0.35
Control group	45	5.09 ± 0.37	4.85 ± 0.31	44.32 ± 0.79	40.81 ± 0.53	92.85 ± 0.75	90.33 ± 0.62
*t*		0.263	8.958	0.296	53.160	0.064	46.828
*P*		0.793	<0.001	0.768	<0.001	0.949	<0.001

## Data Availability

The datasets used during the present study are available from the corresponding author upon reasonable request.
